# Leiomyosarcoma of inferior vena cava involving bilateral renal veins: Surgical challenges and reconstruction with upfront saphenous vein interposition graft for left renal vein outflow

**DOI:** 10.4103/0970-1591.70590

**Published:** 2010

**Authors:** Rishi Nayyar, Sabyasachi Panda, Ashish Saini, Amlesh Seth, Shiv Kumar Chaudhary

**Affiliations:** Department of Urology, All India Institute of Medical Sciences, Ansari Nagar, New Delhi - 110029, India; 1 Department of Cardio-Thoracic and Vascular Surgery, All India Institute of Medical Sciences, Ansari Nagar, New Delhi - 110029, India

**Keywords:** Inferior vena cava, left renal vein ligation, leiomyosarcoma, nephrectomy, renal veins

## Abstract

Leiomyosarcoma of inferior vena cava (IVC) involving bilateral renal veins presents a surgical challenge. Herein, we report the successful management of two such cases using restoration of left renal venous outflow by saphenous vein interposition graft as first step of surgery. Then radical resection of tumor and right kidney was done. IVC was lastly reconstructed using Gore-Tex graft. This report highlights the surgical challenges to ensure radical resection. Furthermore, the importance of restoring left renal outflow in presence of concomitant right nephrectomy is discussed. Both the patients were disease free at six months with no loss of left renal glomerular filtration rate.

## INTRODUCTION

Vascular leiomyosarcomas are rare tumors generally associated with poor prognosis. They form the most common primary tumor type of inferior vena cava (IVC). It was first described by Perl in 1871. Since then, around 300 cases have been reported in the English literature. Aggressive radical resection is the treatment of choice. Following resection, various methods of reconstruction have been described, especially when the tumor involves both renal veins. Ligation of left renal vein is considered to be well tolerated in presence of two functioning kidneys because of collateral pathways. However, in the setting of concomitant right nephrectomy, acute ligation of left renal vein may lead to renal dysfunction and presents a management challenge to preserve as much renal function as possible. Here, we describe a technique of upfront restoration of left renal vein outflow using a saphenous vein interposition graft in two cases. We hypothesize to have preserved maximum possible left renal function using this approach. To our knowledge, no reports of this particular reconstruction have been published for IVC leiomyosarcoma involving renal veins.

## CASE REPORTS

Two cases, one 48-year-old male (Case 1) and another 45-year-old female (Case 2), presented with vague abdominal pain of three and five months duration respectively. The lady also had history of weight loss. Physical examination was normal in both. Imaging included ultrasonography, computed tomography and magnetic resonance imaging, which showed a right retroperitoneal mass arising from inferior vena cava (IVC), invading the right renal hilum and approaching left renal vein ostium [Figure 1]. In Case 2, tumor was extending below to the confluence of common iliac veins. Endovascular biopsy was done in Case 1, but revealed only fibrocollagenous tissue. An informed consent was taken from each case for exploration.

**Figure 1:** MRI TRUFISP coronal images showing IVC tumor (arrow) extending into right vein and infi ltrating right renal hilum. The left renal vein junction with IVC is also involved by the tumor

Exploratory laparotomy was done using a long midline incision. Right colon and small bowel mesentery were reflected to expose the retroperitoneum. The right renal hilum was encased by the tumor. Infra-tumoral IVC or left common iliac vein, left renal vein and supra-tumoral IVC were identified and isolated as first step of surgery. A saphenous vein graft was isolated simultaneously by another team of cardio-thoracic surgeons. The vein was divided into two 12-15 cm segments, each of which was detubularized and then stitched longitudinally to each other [Figure 2] so as to create a wider lumen interposition graft. Vascular side clamps were then placed and the saphenous vein interposition graft was anastomosed between left renal vein and infratumoral IVC (Case 1) or left common iliac vein (Case 2) to provide a passage for continuous drainage of blood from left kidney. This step presumably avoided detrimental effects of acute ligation of left renal vein which was necessary to complete the rest of the procedure. The distal left renal vein, right renal artery and right ureter were then ligated and cut [Figure 2]. The IVC was clamped above and below the tumor which was then resected en bloc with the right kidney. An extended lymphadenectomy of the hilar, paracaval, and interaortocaval lymph nodes was also performed. IVC reconstruction was lastly done using a tube Gore-Tex graft to cover the defect. Total surgical time and blood loss was 290 min and 900 ml in Case 1, and 340 min and 1300 ml in Case 2. There were no post-operative complications and patients had an uneventful recovery. Histopathology confirmed leiomyosarcoma with margins free of tumor.

**Figure 2:** Operative photographs showing (a) Saphenous vein interposition graft (G) placement between left renal vein (LRV) and infratumoral inferior vena cava (IVC) before tumor resection in a case of IVC leiomyosarcoma involving bilateral renal veins. The ligated stump of right renal artery (RRA) is seen over the aorta. The left renal vein stump (LRVS) is also seen over the dilated part of IVC involved by the tumor (T). (b) Final appearance after complete vascular reconstruction. The IVC was reconstructed with a 20-mm wide Gore-Tex graft (GG). (c) Saphenous vein interposition graft formed by longitudinally stitching two detubularized segments of great saphenous vein. (d) Gross specimen

Patency of the saphenous graft was confirmed in both cases with Doppler study at day 3. Anti-coagulant therapy was continued for three months. Pre and post-operative renal function of the left renal unit remained same as confirmed by glomerular filtration rate (GFR) assessment at three months; 54 and 52 ml/min in Case 1 and 46 and 46 ml/min in Case 2. Case 2 also received 600cGy of adjuvant radiotherapy. The cases have completed six and nine months follow up respectively with no evidence of recurrent or metastatic disease on repeat imaging studies.

## DISCUSSION

Vascular leiomyosarcomas are rare tumors arising from the smooth muscle of the vascular media and generally associated with poor prognosis. They constitute 1-2% of all soft tissue sarcomas[1] and form the most common primary tumor of IVC. Depending on location, it can be classified as Type I = infrarenal IVC (36% cases), Type II = renal vessels to retrohepatic IVC (44% cases), and Type III = suprahepatic IVC (20% cases).[2] They are seen predominantly in females (M:F ratio = 1:5) at a mean age of 54 years.[3] Symptoms are usually insidious and nonspecific. Diagnosis is mainly radiological. In equivocal cases, histologic confirmation can be obtained with percutaneous or endovascular biopsy.

Goals of management are to achieve local control, maintain venous return and to prevent recurrence.[4] Aggressive radical resection is the treatment of choice. Following resection of Type II tumor, various methods of reconstruction have been described.[5,6] However, reconstruction of renal venous flow remains debatable. Generally, the ligation of left renal vein is well tolerated in presence of two functioning kidneys because of existence of venous collaterals (lumbar, gonadal and adrenal veins). However, data in the setting of concomitant right nephrectomy is scant and conflicting. Renal dysfunction has been reported after acute ligation of left renal vein by several authors.[7–9] Conversely, others have reported full recovery of renal function after a brief period of anuria.[10] In a recent review, Brian *et al*.[11] suggested the need of left renal vein reconstruction in patients with a solitary left kidney, preoperative renal insufficiency or for resections that will endanger existing collaterals. We believe acute ligation of left renal vein does add to loss of renal function, particularly in the setting of tumor causing only partial luminal block of the left renal vein as was seen in these two cases. This is because the collateral flow is not tuned to high blood flow from the kidney. As against this, if left renal vein is already obstructed completely by the tumor, usually the collaterals have had enough time to dilate and take over the function of draining the left kidney. On the basis of this hypothesis, we believe to have preserved maximum possible renal function in these cases using technique of upfront restoration of left renal vein outflow with saphenous vein interposition graft. Indeed, pre and post-operative GFR confirm to these assumptions. To our knowledge, no reports of this particular reconstruction have earlier been published.

Following resection, management of IVC is also controversial. Reconstruction is preferred over ligation because thrombus may form in the blind end and extend above the hepatic vein causing Budd-Chiari syndrome. Different methods of IVC reconstruction are simple repair, patch repair (using pleura, pericardium, and rectus sheath) and segmental replacement using autologous vein or prosthetic materials like Dacron, PTFE, Gore-Tex, or Teflon. The indication and duration of anticoagulation prophylaxis or adjuvant therapy are also debatable given the rarity of disease. Role of chemotherapy is poorly defined with no documented consistent advantage seen with it.[12] Adjuvant radiotherapy has shown decrease in local recurrence rate by 35%,[4] but its dose is not standardized. We used adjuvant radiotherapy in Case 2 because of extensive involvement and fear of residual tumor in the retroperitoneum. Perioperative mortality ranges between 0 and 15% with 5 and 10 year survival rates of 49.4 and 29.5% respectively.[2] Local tumor recurrence rate may be as high as 57.3%.[4] Poor prognostic factors are upper IVC segment involvement, lower limb edema, Budd-Chiari syndrome, intraluminal tumor growth, and IVC occlusion.[2]

In conclusion, management of IVC leiomyosarcoma involving bilateral renal veins remains a surgical challenge. Left renal venous outflow reconstruction may avoid possible ischemic nephropathy and help preserve maximum renal function. It should especially be considered in presence of concomitant right nephrectomy. Such tumors require highly specialized tertiary centers with expertise in vascular, urologic and oncological surgery.
